# Application Analysis of Radial Basis Function Neural Network Algorithm of Genetic Algorithm for Environmental Restoration and Treatment Effect Evaluation of Decommissioned Uranium Tailings Ponds

**DOI:** 10.1155/2021/1650096

**Published:** 2021-11-24

**Authors:** Kun Wei, Guokai Xiong, Zhenghua Xu, Yong Liu

**Affiliations:** ^1^School of Resource Environment and Safety Engineering, University of South China, Hengyang 421001, Hunan, China; ^2^Decommissioning Engineering Technology Research Center of Hunan Province Uranium Tailings Reservoir, University of South China, Hengyang 421001, Hunan, China; ^3^Hunan Provincial Key Laboratory of Emergency Safety Technology and Equipment for Nuclear Facilities, Hengyang 421001, Hunan, China

## Abstract

A new analysis method for the environmental stability of uranium tailing ponds is established in this paper, and the stability intervals and environmental stability rates of indicators are defined in precise mathematical language and analyzed with examples. The results show that the overall environmental stability of this uranium tailings pond is still in a poor state after the first phase of decommissioning treatment, and special decommissioning treatment should be carried out for factors such as pH and radionuclides Po and Pb. Using the powerful nonlinear mapping function of the artificial neural network, a radial basis function neural network algorithm was constructed to predict the environmental stability of the uranium tailing pond. It provides a new feasible method for the comprehensive evaluation technology of uranium tailings ponds. *Accuracy in DOA Estimation*. The research work in this paper mainly analyzed the environmental stabilization process and stability of decommissioned uranium tailings ponds, proposed a new concept of environmental stability with ecological and environmental protection concepts and gave it a new connotation, established an environmental stability evaluation index system for decommissioned uranium tailings ponds through index screening by using rough set theory, comprehensively considered the influence of environmental factors such as external wastewater and exhaust gas, and realized the multifactor. The system of evaluation indexes for the stability of decommissioned uranium tailings ponds was established by combining multiple factors, and the long-term monitoring and modeling of the environmental stabilization process of decommissioned uranium tailings ponds was carried out by using mathematical methods. The results show that the RBFNN-GA algorithm can reduce the training error of the random radial basis function neural network, improve the generalization ability of the network, and make it capable of handling large data sets.

## 1. Introduction

The goal for the governance and management of uranium metallurgical tailings is that the decommissioning environment must be restored to an acceptable level that allows for the protection of present and future personnel and the environment, with considerations for future generations that include potential radiation exposure, economic consequences, and requirements for monitoring and maintenance, and that do not place an undue burden on future generations. However, the current concept of stabilization of tailings ponds in China only considers their mechanical properties and uses only the mechanical stability of tailings dams as a criterion for judging the safety or otherwise of uranium tailings ponds, which obviously can no longer meet the needs of ecological and environmental protection and sustainable development of uranium tailings pond decommissioning management [1]. From the perspective of protecting the ecological environment and safeguarding the safety of public life and property, it is of great significance to analyze and study the stabilization process and stable state of decommissioned uranium tailings ponds [2]. Therefore, it can better reflect the objective existence of ambiguity. For uranium tailings ponds, due to the complex environmental factors, how to define the stability of various environmental monitoring indicators and the overall stability of the environment is itself a difficult problem to determine. However, the current analysis and evaluation of the stability of uranium tailing ponds only consider the mechanical stability of tailings dams, and only the mechanical stability index of tailing pond dams as the evaluation index of the safety of decommissioned uranium tailing ponds obviously cannot meet the needs of ecological environmental protection and sustainable development of decommissioned uranium tailing ponds. In this paper, based on the systematic examination of the factors influencing the environmental stability of uranium tailings ponds, the analysis of the change pattern of environmental monitoring items of uranium tailings ponds over time, the analysis of the environmental stabilization process characterization of uranium tailings ponds, a new concept and connotation of the environmental stability of uranium tailings ponds in a comprehensive and systematic way, the establishment of the environmental stability evaluation index system of decommissioned uranium tailings ponds were proposed [3]. The analysis method of environmental stability of tailings was constructed, and the quantitative calculation of environmental stability rate was carried out, and the environmental stability grade of each month was divided, on this basis, the environmental stability of existing decommissioned uranium tailings ponds was evaluated and predicted, and a new method of environmental stability analysis and prediction of decommissioned uranium tailings ponds was systematically established, which further enriched and improved the comprehensive evaluation technology of decommissioned uranium tailings ponds, and has a positive impact. It has positive significance and impact on the decommissioning management and environmental protection of uranium tailings ponds [4].

It is generally believed that uranium mining and metallurgical tailings ponds do not cause great impact on the environment after decommissioning and treatment according to the design, but with the passage of time, influenced by external factors (including earthquakes, rainfall and human damage, etc.), the possibility and infiltration of radionuclides from uranium mine tailings ponds into the reservoir area and mine groundwater through the bottom and dam of the reservoir increases greatly with the growth of its age and the infiltration of radionuclides from the groundwater in the reservoir, causing pollution of the reservoir area and mine water environment, which then spreads to various organisms in the biosphere and causes serious ecological hazards, and this hazard has the characteristics of long-lasting, hidden, large degree of harm and difficult to repair; based on the above problems of decommissioned uranium tailings ponds, the effect of treatment in the end needs to be scientifically assessed [5]. With time, some uranium metallurgical tailings ponds are inadequately monitored for safety and ineffective after decommissioning treatment. The leakage of toxic pollutants from uranium tailings dams in the nuclear industry can cause serious accidents, will have a significant impact on the natural environment, and negatively affect the safety of the living environment, and with the migration of radioactive elements, the impact will be further expanded and is difficult to recover. Therefore, strengthening the safety supervision of uranium tailings dams, the treatment of pollutants in uranium tailings dams, and the scientific assessment of the treatment effect are of great practical importance to help people understand the current situation of uranium tailings dams and the treatment effect and to inform people about the safety of nuclear production and social and environmental safety.

At present, there is no clear regulation and management for the effect of management of uranium mine tailings ponds after decommissioning in China, which leads to the lack of clarity of environmental protection departments at all levels on the issue of the effect of management of uranium mine tailings ponds after decommissioning, and the management of uranium mine tailings ponds after decommissioning is a comprehensive work, involving safety supervision, environmental protection, and many other departments. Only a scientific assessment of the effectiveness of the current situation of the tailing's ponds can improve their shortcomings and defects, improve the effectiveness of governance, and ensure the stability of the environmental impact of the uranium mine tailings ponds after decommissioning, which is of great significance to ensure the safety of people's lives and health. The environmental management of uranium tailings ponds is only based on whether the monitoring values of each item meet the standards; i.e., it is usually considered safe to be lower than the emission standards and unsafe to be higher than the emission standards; however, due to the special nature of uranium tailings ponds themselves, their surroundings are easily affected by various factors such as rainfall, earthquakes, dam structure, and human intervention, and the data obtained from monitoring at different moments often vary greatly. We perform 30 trials on each training set and test set and then take the median as the result to reduce the impact of random errors. The stabilization process of each environmental indicator needs to be considered comprehensively to make an objective and effective analysis and evaluation of the environmental stability state of uranium tailings ponds.

## 2. Status of Research

Uranium tailings ponds, as a major hazard source and a long-term potential source of huge radioactive pollution, are ranked 18th in the international ranking of disaster accidents, in which radionuclides, heavy metals, and other toxic and hazardous substances have caused serious pollution to the ecological environment around the tailings ponds through diffusion and migration, posing a serious threat to the safety of downstream residents and facilities, and the quality of their environment is increasingly becoming a concern [6]. Because of the current research status of uranium tailings ponds and related problems of stability research, the author summarized the current research status of environmental stability analysis of uranium tailings ponds at home and abroad by reading a large amount of relevant literature on safety, environment, and stability of uranium tailings ponds at home and abroad [7]. It is important to focus on the three aspects of tailings dam seepage stability analysis, stability analysis of tailings dam deformation and mechanical characteristics, and comprehensive evaluation of uranium tailings pond environment [8]. The analysis methods for tailings dam stability mainly include numerical analysis method and limit equilibrium analysis method, the numerical analysis method is only applied to theoretical discussion and analysis, while the limit equilibrium method is more used in engineering practice; the comprehensive evaluation of the environment mainly applies fuzzy comprehensive evaluation, artificial neural network evaluation, and grey comprehensive evaluation methods [9]. Since radioactive waste is both radiation hazardous and chemically toxic, the treatment of uranium tailings should provide an acceptable level of environmental protection and must provide an acceptable level of human health protection, ensuring that it is within the limits set by the state and predicting that the impact of uranium mining and metallurgical facilities and radioactive waste treatment on the health of future generations is below the dose level of the relevant standards [10]. The residual uranium, needles, radium, etc. and decay substrates in uranium tailings have half-lives of several years, decades, centuries, or even tens of thousands of years and will have a long period of radioactive and chemical hazards to the surrounding atmosphere, water bodies, soil, vegetation, and other apparent environments, groundwater, and organisms, etc. Therefore, the decommissioning treatment of uranium tailings should adopt advanced technologies and methods, appropriate safety, and control measures as far as possible, to ensure that the treatment of uranium tailings the measures should be sufficiently stable and safe for a long period [11].

The environmental performance assessment method is now mainly applied to enterprise environmental performance, which mainly refers to the main achievements and effects achieved by enterprises in their business activities, due to environmental protection and management of environmental pollution; generally speaking, enterprise performance refers to the economic benefits of enterprises, comprehensive hierarchical analysis, and principal component analysis to build an index system to systematically assess the economic performance or environmental performance [12]. An assessment method in the systematic assessment and theoretical assessment results are more objective; the system construction is also more flexible; the disadvantage is that the implementation of a certain degree of difficulty requires a certain theoretical basis and scientific research capabilities to build the index system and determine the assessment scheme. In the stability study of tailings dam deformation and mechanical characteristics, the stability analysis is mainly carried out using the limit equilibrium method [13]. Taking the tailings pond in Hunan Province as an example, the influence of tailings and its medium parameters on the stability and dynamic response of the tailings pond was analyzed by a combination of numerical simulation and model test, and the characteristics and laws of the seismic dynamic response of the tailings pond were summarized systematically by static analysis and dynamic calculation [14]. Baghaee et al. introduced the reliability theory into the stability of tailings dams based on the limit equilibrium theory and the traditional safety factor method. The feasibility and effectiveness of this method were verified [15]. The stability of tailings dams was analyzed based on the finite element method using ANSYS software, which verified the significant advantages of the numerical method in the stability calculation of tailings dams and effectively reflected the stability of tailings dam, providing a certain basis for the safety management of tailings ponds. The stability of the tailings pond accumulation dam was analyzed by using the circular arc bar division method, and the safety coefficient of the dam was calculated by the mechanical geometric model, which effectively reflects the current situation of the tailings dam stability. A three-dimensional numerical simulation study of the tailings dam was carried out using FLAC3D software, and the stress distribution laws of the tailings dam deformation were derived.

Based on the environmental monitoring data of uranium tailing ponds, the dynamic change pattern of environmental indicators over time was systematically analyzed, and the decommissioning management situation and stabilization trend of each environmental monitoring item were initially analyzed. The environmental stability evaluation index system of decommissioned uranium tailing ponds was constructed by considering three aspects, namely, external seepage water, atmospheric environment, and radioactive pollution, and the core index system of comprehensive environmental stability evaluation was finally determined by applying the method of rough set attribute simplification for index screening; the weights of each evaluation index were determined by using the GO method to construct a judgment matrix, and the stability grade of uranium tailing ponds was determined according to the weighted average principle. The environmental stability prediction model based on the BP neural network was established to predict the environmental stability rate and stability grade of a decommissioned uranium tailing pond by using its powerful nonlinear mapping function, and the prediction results were in good agreement with the actual situation.

## 3. Analysis of Radial Basis Function Neural Network Algorithm with Genetic Algorithm for Environmental Restoration and Treatment Effectiveness Evaluation of Decommissioned Uranium Tailings Ponds

### 3.1. Radial Basis Function Neural Network Algorithm Design for Genetic Algorithm

Most of the existing neural networks are improved in structural design and parameter training; the more complex the structure, the more parameters are often required and the more demanding the correction algorithm. The radial basis (RBF) neural network has been chosen and widely used by most scholars because of its simple structure and its ability to approximate arbitrary nonlinear functions. RBF neural network is a novel and effective feedforward neural network with the best approximation and global optimum performance. RBF neural network is proposed based on the feature that neuronal cells in the human brain have a local response, which simulates the local tuning in the human brain. The generalization situation is also very good, and the generalization results are basically consistent with the test set data. It shows that the results of the random radial basis function neural network in the classification task are also satisfactory. The RBF neural network is a local approximation neural network structure with local tuning and mutual coverage of the receptive domain. The activation function is a radial basis function with multivariate interpolation, and the training method is fast and easy, without the problem of local optimality, which makes RBF neural networks have a wide range of applications in many fields, such as function approximation, classification, pattern recognition, regression problems, and prediction and signal processing. Structurally, RBF neural network has a simple topology and a simple and clear learning and training process [16]. It uses the radial basis function as the activation function, and the nodes in the hidden layer produce a larger output only when the input signal is near the center of the radial basis function. The RBF neural network consists of three layers: the input layer, the hidden layer, and the output layer. There is no weight connection between the input layer to the hidden layer, and the input vector is mapped directly to the hidden layer. The mapping from the input layer to the hidden layer is nonlinear; i.e., the transformation function of the hidden layer is nonlinear. There are connection weights between the implicit layer and the output layer, and the mapping from the implicit layer to the output layer is linear; i.e., the output of the entire network is a linear weighted sum of the outputs of the implicit layer. The topology diagram with structural RBF neural network is shown in Figure 1.

This layer is mainly to pass the input samples to the hidden layer. Before that, data normalization, such as normalization, needs to be done on the input samples so that the input values of each node are in the same order of magnitude to avoid the effect of magnitude. The second layer is the hidden layer, the number of neurons in the hidden layer *J* varies with the application to be solved, and the activation function of each hidden node uses a radial basis function. The radial basis function is a nonnegative nonlinear function that is symmetric about the centroid and decays radially, which has a local response function. The implicit layer performs a nonlinear transformation of the input vector to map the low-dimensional input vector into the high-dimensional space, where it solves problems that would otherwise be unsolvable in the low-dimensional space.

(1) $$\begin{array}{c} h_{j}\left(X\right)=\varphi \left(\frac{\left\|X-c_{i}\right\|}{\sigma_{j}}\right),\\ y_{k}=\sum_{j=1}^{J}w_{ik}h_{j}\left(X\right). \end{array}$$

The main difference between RBF neural networks and other feedforward neural networks is the hidden layer. The “base” of the implicit layer space is a radial basis function so that once the center of the radial basis function of each implicit layer node is determined, the input vector can be mapped to the implicit layer space without the need to connect through weights. The diversity of neural networks is reflected not only in the network model determined by the number of nodes in the hidden layer but also in the radial basis functions selected. The radial basis function of the RBF network is nonlinear, and there are many parameters to be set in the process of building the RBF neural network model, including the center and width of the radial basis function and the connection weights of the connection layer. Moreover, solving the outer weight of the random radial basis function neural network by the least square method is a linear operation, and it is very fast in the calculation. Compared with solving the center and smoothing factor of the neural network through supervised learning, this method can effectively improve the learning efficiency of the network. The choice of the center and width of the radial basis function seriously affects the performance of the RBF neural network [17]. At the early stage of the development of RBF, many scholars have incorporated many optimization algorithms for the parameter optimization of RBF neural networks. It was found that once the center and width of RBF were determined, the RBF neural network became a linear system of equations about the connection weights from the input to the output, at which time the connection weights of the output layer could be obtained by solving with the least-squares method or by training with gradient algorithms such as the gradient descent method. How to select the center and what training weight method to use became the research direction of many scholars on RBF network learning.

(2) $$\begin{array}{c} p_{K}\left(f,f_{wn}\right)=\sqrt{\int_{K}{\left[f\left(x\right)-f_{wn}\left(x\right)\right]}^{2}\text{d}x,}\\ h_{x}\left(y,\theta \right)=g\left\{\theta \cdot \left[x+y\right]\cdot \left(x-y\right)\right\}\prod_{i=1}^{m}\sqrt{\theta_{j}}. \end{array}$$

To explore the function approximation ability of the random radial basis function neural network, the thought method of convergence proof of random weighted feedforward neural network is applied to prove that the random radial basis function neural network can approximate any continuous function. The convergence error between the stochastic radial basis function neural network and the approximated function can be known from the analysis process. As the number of neuron nodes *n* increases, the convergence error gradually decreases tending to 0. It is easy to reach the error range that one can accept, so the neural network is an efficient function approximator. The work has shown theoretically that the stochastic radial basis function neural network is capable of approximating arbitrary continuous functions and is also an efficient function approximator. To verify the above theoretical results, we give algorithms on how to solve for the weights of the output layer of the stochastic radial basis function neural network.

(3) $$\begin{array}{c} t_{j}=\sum_{i}^{m}\beta_{i}g\left(\frac{\left\|X_{i}+y_{j}\right\|}{\varsigma_{i}^{2}}\right),\\ H=\left[\begin{array}{ccc} g\left(\frac{{\left\|X_{i}+y_{j}\right\|}^{1}}{\varsigma_{i}^{2}}\right) & ... & g\left(\frac{{\left\|X_{i}+y_{j}\right\|}^{3}}{\varsigma_{i}^{2}}\right)\\ ... & ... & ...\\ g\left(\frac{{\left\|X_{i}+y_{j}\right\|}^{2}}{\varsigma_{i}^{2}}\right) & ... & g\left(\frac{{\left\|X_{i}+y_{j}\right\|}^{5}}{\varsigma_{i}^{2}}\right) \end{array}\right]. \end{array}$$

This idea has been used in several studies, such as the introduction of kernel methods for data classification in over-the-limit learning machines and stacked kernel networks (SKNs). However, a neural network model of the class of overdetermined learning machines, which essentially solves for a stochastic suboptimal solution of the network, is difficult to achieve the same results in large data. Stacked kernel networks, on the other hand, successfully apply kernel methods to classification tasks but also point out that the use of kernel methods can easily lead to overparameterization and overfit the network. Therefore, the introduction of kernel methods into deep learning models requires further exploration (Figure 2).

Therefore, instead of using these two ways of introducing kernel functions, this topic uses the ordinary radial base layer. Although this weakens the role of the kernel method, this cuts down the number of parameters in the model and makes it easier to avoid the problem of model overfitting due to overparameterization. In addition to the background related to the kernel method, the Gaussian function's properties are also of interest. In this way, the order of things based on the comparison feature is determined by the comparison result of a certain feature, and the order obtained from this comparison is used to judge the general situation of the membership function of these things for the specific feature, and then, the membership function is further constructed. To solve, the binary comparison ranking method is different according to the contrast measure. For example, the local approximation property, where the parameters associated with a local target space are only a small fraction of the total parameters, also fits some mechanisms of the organism. In terms of the mathematical nature of the function, the target of activation is not the data itself but the distance of the data from a particular central vector, and the fact that Gaussian functions have infinite order derivatives is also an advantage [18]. As a result, this topic proposes a radial basis self-encoder model, which consists of an input layer, a radial basis kernel function layer, and a self-coding layer, which is an improvement of the self-classical self-encoder model. Mathematically, in essence, the process of solving the model parameters is to solve the optimization problem shown in equation (4), which is often nonconvex, so it is important to choose a suitable solution. In this topic, we will combine the properties of Gaussian functions and use a gradient-based optimization algorithm for the parameter solution.

(4) $$\begin{array}{c} \theta^{*}=\arg\max L\left(\theta^{2},x_{1},g^{2}\left(f\left(\phi \left(X\right)\right)\right)\right). \end{array}$$

Like the classical self-encoder model, the training of the radial-based self-encoder model proposed in this paper also employs a back-propagation algorithm and uses a gradient-based training method. The data first go through a forward propagation process to get the output under the current model parameters, then, some loss function is used to measure the deviation of the current output from the true value, and then, the current model parameters are corrected and the next calculation is performed through a backward propagation process, and such an iterative process continues until a specific condition is satisfied and terminated. In this topic, the Gaussian function is chosen as the activation function for the radial basis function layer, and since the Gaussian function contains two hyperparameters center vector and variance, which can be selected in various ways, this section will discuss the methods for selecting these two hyperparameters as well as the overall network optimization methods (including loss function selection, activation function selection for the classical layer, and gradient-based methods for overall network parameter optimization).

### 3.2. Experimental Design for the Evaluation of Environmental Restoration and Treatment Effects of Decommissioned Uranium Tailings Ponds

ISO 14001 is the number of environmental management systems certified by the International Organization for Standardization. It is a standard developed in response to the global environmental damage and environmental pollution that is becoming more and more serious, global warming, destruction of the ozone layer, reduction of biodiversity, and other major ecological and environmental problems that threaten the future survival and sustainable development of mankind, to comply with the development of international environmental protection, to take the road to sustainable development, and following the needs of international economic and trade development. ISO 14001 states that environmental performance is the measurable effectiveness of an organization's environmental management system based on environmental policies, objectives, and targets to control its environmental factors. The “organization” is the actor, which can be either a company or a government (department). The source of environmental performance varies from subject to subject [19]. Depending on the source of environmental performance, environmental performance is divided into organizational environmental performance and regional environmental performance.

Some scholars define environmental performance as an evaluation indicator of production efficiency that takes environmental issues into account and is used to analyze some of the problems of economic development in harmony with the environment, with its meaning being mainly the ratio of the economic value of products and services that meet human needs to the environmental load, i.e., the corresponding economic benefit per unit of environmental impact. The definition states that to improve environmental performance, people must take the initiative to control environmental pollution and protect the environment while carrying out development. Through the scientific and reasonable evaluation of the environmental efficiency of enterprises, individuals, or related organizations in the work of environmental management assessment, we can find out some necessary links between the situation of environmental protection and economic growth and some key problems of mutual constraints and influences between the two, to further provide new reference basis for managers or plan makers and then on a certain basis to revise. Obviously, it has been unable to meet the needs of ecological environment protection and sustainable development for the decommissioning of uranium tailings ponds. Whether it is from the perspective of protecting the ecological environment or protecting the safety of public life and property, the analysis and research on the stabilization process and stability status of decommissioned uranium tailings ponds are of great research significance. Therefore, environmental performance assessment is a rather important way and assessment tool for individuals, enterprises, institutions, and projects, as shown in Figure 3.

As a systematic process for assessing and measuring environmental performance in all aspects of an organization's internal economy, environmental performance assessment provides a reliable and optimal guide for program design and implementation of economic investments, etc. within an organization. The process includes the selection of parameters, data collection and statistical analysis, information evaluation based on environmental performance guidelines, evaluation reports, and academic communication, and targeted periodic review and improvement of the evaluation process. As an internal implementation process and management tool, the purpose of environmental performance assessment is to provide managers with reliable and verifiable external environmental information of varying relevance to assess the gaps and shortcomings between an organization's environmental performance and the standards set by the organization's managers and to make further improvements and optimizations [20]. In the whole process of collecting and evaluating information, environmental performance assessment has a clear continuous (including past, present, and future) character compared to other methods. The purpose of environmental performance assessment is to provide a detailed description of the strengths and weaknesses of environmental conditions, to reveal the overall situation of environmental policies and environmental changes, to significantly improve the environmental awareness of all sectors of society, and to scientifically measure the level of management of organizations and their environmental managers. A sound environmental performance assessment is a prerequisite for the objective and effective management of organizations and projects.

The concept of stabilization of uranium tailings ponds only considers their mechanical properties, and only the mechanical stability index of tailings ponds as the evaluation index of the safety of decommissioned uranium tailings ponds can no longer meet the needs of ecological environmental protection and sustainable development of decommissioned uranium tailings ponds. The concept and connotation of environmental stabilization of decommissioned uranium tailings ponds proposed in this paper objectively reflect the necessity of evaluating the environmental stability of decommissioned uranium tailings ponds, which requires comprehensive consideration of environmental radiation, effluents, and other factors, to establish a reasonable evaluation index system, which is also the key to the evaluation of the stability of decommissioned uranium tailings ponds. The evaluation index system should be based on a system perspective, on the one hand, to grasp the key factors, and on the other hand to consider all other factors, so that the evaluation index system can reflect the actual situation of the evaluated object comprehensively and objectively. For the uranium tailings pond system, the index system should comprehensively include seepage water environmental indicators, atmospheric environmental indicators, and radiation environmental indicators (Figure 4).

The number of indicators in the indicator system should be reduced as much as possible, and the core impact indicators should be highlighted, so as not to make the evaluation indicator system too large and affect the accuracy of the evaluation results, and to avoid the interrelationship between indicators so that the selection of indicators is both adequate and necessary. For uranium tailing ponds, on the premise of including the main environmental monitoring indicators and the indicators with greater impact on the environment of uranium tailing ponds, irrelevant or harmless environmental indicators should be reduced as much as possible. The indicator system is used to describe social phenomena, and science is the premise and basis for the existence of the indicator system. Therefore, it is necessary to start from the actual situation, and the constructed indicator system should be able to objectively reflect the actual situation, while the indicators included should be in line with the scientific and theoretical basis. The uranium tailings pond is a complex system, and the indicator system should be able to analyze and compare with existing theories and methods, while the indicators with inclusive relationships should be deleted appropriately, and cross-over information should be avoided between each layer of indicators [21]. The process of constructing the indicator system is essentially the process of decomposing the top target layer by layer, so the evaluation indicator system is also a multilayer and multi-indicator system, analyzing the complex evaluation problems layer by layer, considering them comprehensively, grasping the key points, and considering both qualitative and quantitative indicators. Through the analysis of the change law of the environmental monitoring project of uranium tailings pond over time, the characterization of the environmental stabilization process of the uranium tailing pond is analyzed, and the new concept and connotation of the environmental stability of the uranium tailing pond are comprehensively and systematically put forward. There is an environmental stability evaluation index system for decommissioned uranium tailings ponds. According to the actual situation of uranium tailings ponds, the environmental indicator system can usually be decomposed into three levels, and the decomposition process is from coarse to fine, from macro and micro, and from general to specific.

Fuzzy mathematics takes uncertainty as its research object; it uses precise mathematical language to describe fuzzy phenomena, so it can better reflect the objective fuzzy phenomena. For uranium tailings ponds, because of the complex environmental factors, how to define the stability of each environmental monitoring index and the comprehensive stability of the environment is itself a difficult problem to determine, and the use of fuzzy mathematical theory can make up for the shortcomings of exact mathematics and stochastic mathematics by making the fuzzy objects exact. In fuzzy mathematics, there are many branches such as fuzzy topology, fuzzy group theory, fuzzy graph theory, fuzzy probability theory, fuzzy linguistics, and fuzzy logic. After decades of development, they have been widely used in many neighborhoods. This thesis is theoretically feasible to use fuzzy mathematical theory to analyze the environmental stability of uranium tailing ponds.

## 4. Results and Analysis

### 4.1. Performance Results of Radial Basis Function Neural Network Algorithm with Genetic Algorithm

For these three datasets, we simplify the centroids of the hidden layer neurons in the random radial basis function neural network, and the smoothing factors uniformly distributed between [−1, 1] and [0, 1], respectively. Thirty trials were conducted for each training and test set, and then, the median was taken as the result to reduce the effect due to random errors. The results of the performance test of the random radial basis function neural network are shown in Figure 5. During the task of fitting the cos (z) function of the random radial basis function neural network, the training error becomes smaller and smaller as the number of neuron nodes in the hidden layer gradually increases, and the fitting results become better and better. Observing Figure 5, it can be found that when the number of neuron nodes is small, the fit is inadequate, and as the number of neuron nodes increases, the fitting result of the random radial basis function neural network is gradually able to match the cos (a) function. It should be noted that the fitting results are not the same for each training here because of the random selection of some parameters in the network, and we have selected one of the cases for the graph.

To be able to better represent the performance of the stochastic radial basis function neural network, the Spectra dataset was selected to test its fit. Unlike the dataset with one-dimensional cos (z) functions for both input and output, the Spectra dataset has a higher dimensionality than the actual data. Figure 5 directly illustrates how the training error gradually decreases as the number of hidden layer neuron nodes increases during the fitting of the random radial basis function neural network to the Spectra training set.

The generalization of the random radial basis function neural network on this Spectra test set is also very good, and the generalization results can match the test set data. It illustrates the equally satisfactory results of the random radial basis function neural network in the classification task. In the classification dataset, the recognition rate in its training set can reach almost 100% with the increase of neuron nodes in the hidden layer of the network, and the highest recognition rate in the test set is close to 90%. Observation of the recognition rate in the test set reveals that the curve has a first increase and then decrease, which is because, with the increase of the number of hidden layer nodes, the weights of the output layer of the random radial basis function neural network derived by the simple RBFNN algorithm can easily lead to the overfitting phenomenon of the neural network. From Figure 6, the training time of the random radial basis function neural network is very short in the training tasks of both the Spectra dataset and Iris dataset, reflecting its fast-learning ability. According to the two curves toward the situation, the training time of the neural network increases gradually with the number of neuron nodes. The input dimension of Spectra is 401 dimensions and the output dimension of Iris is 4 dimensions. But the difference in training time between the two is only in the microsecond level, which is enough to show that the random radial basis function neural network has great potential to handle large data set tasks.

The random selection of some parameters in the radial basis function neural network is an important complement to the existing how to determine the radial basis function neural network center and smoothing factor. Improving its shortcomings and deficiencies, improving the governance effect, and ensuring the stability of the environmental impact after the decommissioning of the uranium mining and metallurgical tailings pond are of great significance to ensure the people's life, health, and safety. Unlike traditional BP neural networks, this random setting of radial basis function centers and smoothing factors makes it possible to calculate only one parameter, the output layer weight, in a radial basis function neural network with a three-layer network structure, which drastically reduces the number of parameters to be solved in the network. And solving the stochastic radial basis function neural network outer weights by least squares is a linear operation, which is very fast in computation. Compared to solving the center and smoothing factors of a neural network through supervised learning, taking this approach can effectively improve the learning efficiency of the network, making it a great potential for handling big data tasks. In this paper, we use the properties of generalized functions to construct a limit integral expression for the approximated function; secondly, we use Monte Carlo methods to compute the integrals in this expression and theoretically prove that this random radial basis functions neural network is not only capable of approximating arbitrary continuous functions but also an efficient function approximator. And the random radial basis function neural network is tested by fitting and classifying simulation by selecting different data sets. The results show that the stochastic radial basis function neural network does exhibit good performance.

### 4.2. Results of the Evaluation of the Environmental Rehabilitation and Treatment Effects of Decommissioned Uranium Tailings Ponds

Benchmarking, also known as benchmarking, is a method of environmental performance assessment in which an organization sets itself an example and a goal to strive for in its development process, with the basic idea of systematic optimization, continuous improvement, and continuous improvement. Benchmarking is unique in its assessment method, which is achieved through comparison. The first step in the benchmarking method is to identify a benchmark, usually a leading organization in the field, as a goal for the organization to strive for. At the end of each implementation phase, the results are compared with the identified benchmark, and a phase summary assessment is conducted to adjust the next phase of the approach until finally the benchmark level is reached and a higher benchmark is identified, as shown in Figure 7.

The binary comparison ordering method is more practical in the method of determining the affiliation function, which is implemented by making a reasonable two-by-two comparison of certain specific features between multiple things, to determine the order of things based on this comparison feature with the comparison result of certain features, and the order obtained from this comparison is used to judge the approximate situation of these things for the affiliation function under this specific feature and further then construct the affiliation function for solving; the binary comparison ranking method can be divided into relative comparison method, comparison average method, priority relationship ordering method, and similar priority comparison method according to different comparison measures, as shown in Figure 8. The RBF neural network was proposed based on the characteristics of the human brain's neuronal cells that have a local response. It simulates the local approximation neural network structure of the human brain that is locally adjusted and covers the receptive domains.

As a result, a large amount of acidic wastewater is generated, which flows through a special pipeline to the wastewater treatment plant, where it is degraded and precipitated so that the heavy metals in it are precipitated and neutralized using lime, and then, the treated wastewater is discharged to the tailings pond. The wastewater migrates from the outfall to each section of the tailings reservoir, and the distance from each dam section to the outfall varies, resulting in different degrees of contamination. Dam B is located at the southwest end of the tailings dam, and due to the distance, the wastewater needs to flow for some time to reach this dam section, so the change in the pH of the water body is relatively flat, and because the wastewater contains more free state ammonia ions. The larger the concentration of ammonia ions, the more *H*+ produced by hydrolysis, and the more severe the acidification of the water body. The variation of pH values with time was plotted based on the monitored raw data. A new method for environmental stability analysis of uranium tailings ponds is proposed, and the stability intervals of indicators and environmental stability rates are defined in precise mathematical language, which is of positive significance for further enriching and improving the comprehensive evaluation techniques of decommissioned uranium tailings ponds.

## 5. Conclusion

The research work in this paper mainly analyzes the environmental stabilization process and stability of decommissioned uranium tailing ponds, proposes a new concept of environmental stability with ecological and environmental protection concept and gives it a new connotation, establishes an evaluation index system of environmental stability of decommissioned uranium tailing ponds through index screening using rough set theory, integrates the influence of environmental factors such as external wastewater and exhaust gas, and realizes the multifactor. The system of evaluation indexes for the stability of decommissioned uranium tailing ponds was established by combining multiple factors; the long-term monitoring and model verification of the environmental stabilization process of decommissioned uranium tailing ponds were carried out by using mathematical methods, and the change law of the stability of environmental parameters over time was studied; the connotation of environmental stability was further deepened and supplemented; uncertainty theories such as statistical theory and fuzzy mathematics were applied to construct a comprehensive evaluation model for the stability of decommissioned uranium. There are an input layer, hidden layer, and output layer. There is no need for a weight connection between the input layer and the hidden layer, and the input vector is directly mapped to the hidden layer. A comprehensive evaluation model of the stability of a decommissioned uranium tailings pond was constructed by applying statistical theory, fuzzy mathematics, and other uncertainty theories, and a prediction model of the environmental stability was established by using BP neural network. The average error rate of the predicted environmental stability rate was only 6.27%. Based on the principle of maximum affiliation, the predicted stability level was the same as the expected stability level of the sample, and the overall prediction results were consistent with the actual situation, which further verified the applicability and feasibility of the method. The degree of influence of environmental indicators on the environmental stability of uranium tailings ponds was also analyzed using the univariate method, which provides a new method and technique for the comprehensive evaluation and decommissioning management of uranium tailings ponds.

## Figures and Tables

**Figure 1:** RBF neural network topology.

**Figure 2:** Flow of constructing safety risk assessment index system for tailing ponds.

**Figure 3:** Statistics on environmental indicators.

**Figure 4:** Technical roadmap for environmental stability analysis and prediction of decommissioned uranium tailings ponds.

**Figure 5:** Results of the function training set fitting.

**Figure 6:** Training error and recognition rate of Spectra dataset under RBFNN algorithm.

**Figure 7:** Classification of environmental performance benchmarking levels.

**Figure 8:** Changes in monitoring values.

## Data Availability

The data used to support the findings of this study are available from the corresponding author upon request.
